The article "Just One Position-Independent Lysine Residue Can Direct MelanA into Proteasomal Degradation following N-Terminal Fusion of Ubiquitin" was published in 2013. Journal: PLoS One.

# Just One Position-Independent Lysine Residue Can Direct MelanA into Proteasomal Degradation following N-Terminal Fusion of Ubiquitin

**DOI:** 10.1371/journal.pone.0055567

**Published:** 2013-02-05

**Authors:** Christian Setz, Melanie Friedrich, Sabine Hahn, Jan Dörrie, Niels Schaft, Gerold Schuler, Ulrich Schubert

**Affiliations:** 1 Institute of Clinical and Molecular Virology, Universitätsklinikum Erlangen, Erlangen, Germany; 2 Department of Dermatology, Universitätsklinikum Erlangen, Erlangen, Germany; Cleveland Clinic Lerner Research Institute, United States of America

## Abstract

N-terminal stable in frame fusion of ubiquitin (Ub) has been shown to target the fusion protein for proteasomal degradation. This pathway, called the Ub fusion degradation (UFD), might also elevate MHC class I (MHC-I) antigen presentation of specific antigens. The UFD, mainly studied on cytosolic proteins, has been described to be mediated by polyubiquitination of specific lysine residues within the fused Ub moiety. Using the well characterized melanoma-specific antigen MelanA as a model protein, we analyzed the requirements of the UFD for ubiquitination and proteasomal degradation of a transmembrane protein. Here we show that fusion of the non-cleavable Ub^G76V^ variant to the N-terminus of MelanA results in rapid proteasomal degradation via the endoplasmic reticulum-associated degradation (ERAD) pathway and, consequently, leads to an increased MHC-I antigen presentation. While lysine residues within Ub are dispensable for these effects, the presence of one single lysine residue, irrespectively of its location along the fusion protein, is sufficient to induce degradation of MelanA. These results show that the ubiquitination, ER to cytosol relocation and proteasomal degradation of a transmembrane protein can be increased by N-terminal fusion of Ub at the presence of at least one, position independent lysine residue. These findings are in contrast to the conventional wisdom concerning the UFD and indicate a new concept to target a protein into the ubiquitin-proteasome system (UPS) and thus for enhanced MHC-I antigen presentation, and might open up new possibilities in the development of tumor vaccines.

## Introduction

The UPS constitutes the main proteolytic system in the cytosol of eukaryotic cells. Ubiquitin (Ub) is attached to Lys, or, in rare cases, other residues [1] of target proteins by the cascade-like catalytic action of E1, E2 and E3 enzymes. Within Ub itself, seven Lys residues can serve as Ub acceptor sites allowing the formation of poly-Ub chains. Monoubiquitination as well as Lys-63-linked polyubiquitination has been shown to regulate cell functions such as DNA repair, signal transduction and endocytosis, whereas polyubiquitination via Lys-48 is the canonical signal for the degradation of the target protein by the 26S proteasome (for review see [2]). The peptides resulting from proteasomal degradation represent the majority of the epitopes that are presented on the cell surface by mature MHC class I (MHC-I) molecules to CD8^+^ T cells [3].

Stable in frame fusion of Ub to the N-terminus of proteins has been shown to augment their proteasomal degradation and thus enhances their MHC-I antigen presentation [4], [5], [6], [7], [8], [9], [10]. The associated proteolytic pathway has been termed Ub fusion degradation pathway (UFD; [5], [6]). Ub fusion proteins can be engineered by mutation of the C-terminal Gly-76 of Ub, which virtually abrogates the removal of the Ub moiety of such UFD fusions by abundant Ub hydrolases [11], [12]. According to current wisdom, the initial step is the attachment of a poly-Ub chain to Lys-48 or -29 of the Ub fusion part, catalyzed by the HECT-type E3 ligase Ufd4 in yeast, or its homologue TRIP12 in mammalian cells [6], [13], [14]. The E4 factor Ufd2 elongates the Ub chain and allows for a better degradation of the UFD substrate by the 26S proteasome [15]. Until now, mostly cytosolic substrates of the UFD pathway have been studied [4], [5], [6], [7], [8]. However, more than 30% of all newly synthesized proteins enter the secretory pathway [16]. Although stable Ub fusion has been described to augment immune recognition of certain transmembrane proteins [9], [10], it has not been analyzed yet if the requirements for ubiquitination of the Ub fusion part in the UFD pathway are identical for cytosolic proteins and substrates that are inserted into cellular membranes.

The accumulation of misfolded proteins in the endoplasmic reticulum (ER) is prevented by a process termed ER-associated degradation (ERAD, [17]). Misfolded proteins are recognized and targeted to one of several ER-resident Ub E3 ligase complexes, which catalyze the polyubiquitination of the substrate at the cytosolic face of the ER membrane [18]. Without any doubt, ERAD substrates need to be retranslocated into the cytosol, in order to become accessible for degradation by the 26S proteasome. The AAA-ATPase (ATPase associated with various cellular activities) valosin containing protein (VCP) is essential for the ATP-dependent extraction of polyubiquitinated proteins from the ER membrane into the cytosol [19], where they are subsequently degraded by the 26S proteasome. Amongst many other functions [20], VCP/p97 has also been shown to be involved in the UFD pathway [21], [22], [23].

To analyze the mechanism of the UFD for a transmembrane protein, we used MelanA (also known as MART-1) as a model protein. MelanA has been discovered as a melanoma-associated antigen targeted by tumor-reactive cytolytic T lymphocytes [24], [25]. It is palmitoylated and localized to the ER as well as transported throughout the Golgi network to become presented at the cell surface [26], [27]. The protein has a luminal N-terminus, followed by a transmembrane domain and an extended C-terminal cytosolic region [27]. Although MelanA has been extensively studied as a target for vaccine development against malignant melanoma, no enzymatic activities or other cellular functions have been yet identified for this membrane protein.

In this study, we demonstrate that stable fusion of Ub^G76V^ to the N-terminus of the transmembrane protein MelanA converted the otherwise stable protein into a substrate for both the UFD and the ERAD pathway, resulting in the rapid proteasomal degradation of the fusion protein. The increased turnover correlated with an enhanced entry into the MHC-I pathway. These effects were, in contrast to the current working model for the UFD, independent of Lys residues within the fused Ub moiety. Both the primary sequence of Ub as well as a position independent single Lys residue in the entire sequence of the fusion protein are sufficient to target MelanA for rapid destruction by the 26S proteasome and thus to enhance its MHC-I antigen presentation. This finding reveals a yet unknown mechanism for the UFD and could be useful in the optimisation of tumor vaccination and augmentation of the immunogenicity of transmembrane antigens.

## Results

### Ub^G76V^MelanA-SL is rapidly degraded by the 26S proteasome and exhibits increased MHC-I antigen presentation

In order to attract the transmembrane protein MelanA into the UFD pathway, Ub^G76V^ was fused to its N-terminus. To analyze if this stable Ub fusion correlates with an enhanced MHC-I antigen presentation of a MelanA-derived epitope, the model epitope SIINFEKL (SL) was introduced as an indicator for antigen processing into the N-terminal region of MelanA and Ub^G76V^MelanA (Fig. 1A).

**Figure 1:** Ub^G76V^MelanA-SL is rapidly degraded by the 26S proteasome and exhibits increased MHC-I antigen presentation. (**A**) Schematic representation of MelanA-SL and Ub^G76V^MelanA-SL proteins. (**B**) After transient transfection, HeLa cells expressing MelanA-SL or Ub^G76V^MelanA-SL were treated with PIs (20 µM MG-132+5 µM LC) or DMSO as a solvent control for 4 h prior to lysis. Whole cell lysates were analyzed by Western blot using an anti-MelanA Ab. As a loading control, the Western blot was reprobed using an anti-β-actin Ab. (**C**) HeLa-K^b^ cells were transiently transfected with expression plasmids coding for MelanA, MelanA-SL or Ub^G76V^MelanA-SL. H2-K^b^-SL complexes presented on the surface of MelanA-positive cells were quantified by flow cytometry using the mAb 25D1.16 conjugated to allophycocyanin (25D1.16-APC). Following fixation and permeabilization, intracellular MelanA was detected by staining with anti-MelanA and a secondary Alexa488-conjugated anti-mouse Ab. A representative histogram plot is shown. (**D**) Depiction of the mean fluorescence intensity (MFI) of the 25D1.16 staining of 36 independent experiments. The statistical analyses were performed using the paired two-tailed student's t-test (_***_p<0.0001). (E) HeLa-K^b^ cells were transiently transfected with expression plasmids coding for MelanA-SL or Ub^G76V^MelanA-SL and qRT-PCR was performed from total RNA. The normalized mRNA amount of MelanA-SL was set to 1 and the mRNA relation of Ub^G76V^MelanA-SL to MelanA-SL is depicted. Bars represent mean ± SD from three independent experiments.

To detect rapidly degraded Ub adducts, a quick cell lysis was performed under conditions where the proteasome and deubiquitinating enzymes (DUBs) were inhibited. When steady-state protein levels in whole cell lysates were analyzed by Western blot using an anti-MelanA Ab, Ub^G76V^MelanA-SL appeared only as a very faint band, while MelanA-SL could be readily detected (Fig. 1B). Following addition of the proteasome inhibitors (PIs) MG-132 and lactacystin (LC) four hours prior to cell lysis, Ub^G76V^MelanA-SL and putative ubiquitinated adducts thereof accumulated (Fig. 1B). This finding indicates a continuous, high turn-over of Ub^G76V^MelanA-SL by the 26S proteasome. As described previously, cleavage of the Ub moiety is greatly impaired, but not completely abrogated by mutation of its C-terminal Gly residue [12], [28]. Therefore, a minor band representing MelanA-SL could be detected in cells expressing Ub^G76V^MelanA-SL (Fig. 1B, lane 4).

To analyze the MHC-I presentation of the MelanA-derived SL-epitope, HeLa cells that stably express the murine SL-binding MHC-I allotype H2-K^b^ [29] were transfected with expression plasmids coding for MelanA-SL or Ub^G76V^MelanA-SL. Flow cytometry analysis using the mAb 25D1.16, which specifically recognizes H2-K^b^-bound SL, revealed that cells expressing Ub^G76V^MelanA-SL displayed higher numbers of H2-K^b^-SL complexes at the cell surface compared to cells expressing the wt protein (Fig. 1C), although the total amount of H2-K^b^ was identical (data not shown). The cumulative results of 36 independent experiments reveal a highly significant two-fold increase in SL-presentation following fusion of Ub^G76V^ to MelanA-SL (Fig. 1D). To exclude that the increased SL-presentation of Ub^G76V^MelanA-SL is due to a higher transcription level of the Ub^G76V^MelanA-SL-encoding plasmid, quantitative RT-PCR experiments were conducted. The quantities of mRNA encoding the wt MelanA-SL and the Ub^G76V^ variant of MelanA-SL were similar (Fig. 1E). Further, to be absolutely sure, we also compared the transfection efficiency by counting the number of MelanA positive cells by FACS analysis that, again, was comparable for both constructs (data not shown). Taken together, these data demonstrate that the stable fusion of Ub to the N-terminus of MelanA-SL results in a rapid proteasomal degradation and an enhanced MHC-I antigen presentation of this transmembrane protein.

### Insertion of SL does not affect the subcellular localization of MelanA

It was previously shown that MelanA is a membrane protein that is predominantly localized in the Golgi network, especially the trans-Golgi network (TGN) [26], [27]. As mislocalization of a protein may enhance its proteasomal degradation [30], [31], we wanted to analyze whether the subcellular localization of MelanA is altered by the insertion of SL or Ub fusion. HeLa cells were transfected with expression plasmids coding for MelanA and MelanA-SL and treated with PIs or DMSO as a solvent control for 4 h. Following fixation, permeabilization and staining with specific Abs, the localization of MelanA and TGN46, a marker for the TGN, was analyzed by confocal microscopy. MelanA accumulated predominantly in a perinuclear compartment and displayed intense colocalization with TGN46. Neither the insertion of SL nor treatment with PIs had any influence on the subcellular distribution of MelanA (Fig. 2A+B).

**Figure 2:** Insertion of SL does not affect the subcellular localization of MelanA. Following transient transfection HeLa cells expressing MelanA or MelanA-SL were treated with (**A**) DMSO as a solvent control or (**B**) PIs (20 µM MG-132+5 µM LC) for 4 h. Cells were stained for MelanA (green) with an anti-MelanA Ab and for TGN using an anti-TGN46 Ab (red). The nucleus was illuminated with DAPI (blue). (**C**) Following transient transfection HeLa cells expressing MelanA-SL or Ub^G76V^MelanA-SL were treated with PIs or DMSO for 4 h. The plasma membrane was permeabilized using 20 µM digitonin followed by a cell fractionation (S = supernatant; P = pellet) and analyzed by Western blot. Staining for the ER-resident protein calnexin served as a control for the quality of the fractionation. As a loading control, the Western blot was reprobed using an anti-β-actin Ab. (**D**) After transient transfection HeLa cells expressing MelanA-SL or Ub^G76V^MelanA-SL were treated with PIs or DMSO for 4 h. The ER fraction was isolated using an ER isolation kit and analyzed by Western blot. Staining for the ER-resident protein calnexin served as a positive control and Hsp90 as a negative control to assess the quality of the fractionation.

To confirm that Ub^G76V^MelanA-SL is still inserted within intracellular membranes and not degraded because of a mislocalization [30], subcellular fractioning analyses following cell lysis using 20 µM digitonin, which selectively perforates the plasma membrane [32], were conducted. After proteasome shutdown, a fraction of Ub^G76V^MelanA-SL and ubiquitinated species thereof became clearly detectable in the pellet fraction, showing that this protein is indeed inserted within cellular membranes. Another fraction of Ub^G76V^MelanA-SL however accumulates in the soluble, cytosolic fraction (Fig. 2C). Staining with the specific ER marker calnexin illustrates the purity of the pellet and the soluble fraction, as calnexin is only detectable in the pellet fraction. To further characterize the localization of Ub^G76V^MelanA-SL within the cell, we specifically isolated the ER resident proteins using a standard system. MelanA-SL as well as Ub^G76V^MelanA-SL were clearly detectable in the ER fraction after proteasome shut down as shown by Western blot (Fig. 2D). The purity of the ER fraction was controlled by different protein markers. Calnexin as an ER marker, but not Hsp90, marker for the cytosol, could be detected in the Western blot (Fig. 2D).

Taken together, these results indicate that the insertion of SL, as well as the stable fusion of ubiquitin to the N-terminus of MelanA, had no influence on its insertion within the ER membrane and the subcellular distribution of MelanA.

### The enhanced proteasomal degradation and MHC-I antigen presentation of Ub^G76V^MelanA-SL are independent of the Lys residues within the fused Ub^G76V^

The stable N-terminal fusion of Ub^G76V^ has been shown to result in the polyubiquitination of Lys residues 48 (K48) or 29 (K29) within the fused Ub moiety [6]. Surprisingly, mutation of K48 or K29 to Arg in the context of Ub^G76V^MelanA-SL had no influence on its metabolic stability or MHC-I antigen presentation (data not shown). Moreover, none of the individual Lys residues within the fused Ub^G76V^ (K6, K11, K27, K33, K63) was essential for the rapid proteasomal degradation or enhanced MHC-I antigen presentation of Ub^G76V^MelanA-SL (data not shown).

Intriguingly, when all seven Lys residues within the fused Ub^G76V^ were exchanged for Arg, this mutant, called Ub^G76V(K0)^MelanA-SL, was still efficiently degraded by the 26S proteasome, preventing its accumulation to detectable levels (Fig. 3A). Similarly to Ub^G76V^MelanA-SL, Ub^G76V(K0)^MelanA-SL as well as putative ubiquitinated species thereof could be detected after addition of PIs (Fig. 3A).

**Figure 3:** The enhanced proteasomal degradation and MHC-I antigen presentation of Ub^G76V^MelanA-SL are independent of the Lys residues within the fused Ub^G76V^. (**A**) Following transient transfection HeLa cells expressing MelanA-SL, Ub^G76V^MelanA-SL or Ub^G76V(K0)^MelanA-SL were treated with PIs or DMSO for 4 h. Whole cell lysates were analyzed by Western blot. As a loading control, the Western blot was reprobed using an anti-β-actin Ab. (**B**) Immunoprecipitation (IP) of ubiquitinated MelanA-SL species. After transient transfection, MelanA-SL and variants thereof were coexpressed with HA- tagged Ub. MelanA was precipitated under denaturing conditions from whole cell lysates using an anti-MelanA Ab. Ubiquitinated MelanA was detected by an anti-HA Western blot. To demonstrate that equal amounts of MelanA and variants thereof are used in the IP, a part of the cell lysate was collected before the IP and stained with an anti-MelanA Ab. As a loading control, the Western blot was reprobed using an anti-β-actin Ab (upper panels). (**C**) Following transient transfection of HeLa-K^b^ cells with MelanA-SL, Ub^G76V^MelanA-SL or Ub^G76V(K0)^MelanA-SL, H2-K^b^-SL complexes presented on the surface of MelanA-positive cells were quantified by flow cytometry using 25D1.16-APC. A representative histogram plot is shown. (**D**) Depiction of the mean fluorescence intensity (MFI) of the 25D1.16 staining of 36 independent experiments. The statistical analysis was performed using the paired two-tailed student's t-test (_***_ p<0.0001).

To confirm that the MelanA species between ∼30 and 43 kDa represent ubiquitinated species of MelanA-SL, N-terminally HA-tagged Ub (HA-Ub) was coexpressed with MelanA-SL, Ub^G76V^MelanA-SL or Ub^G76V(K0)^MelanA-SL in HeLa cells. MelanA-SL was immunoprecipitated from denatured cell lysates using an anti-MelanA Ab, and ubiquitinated species thereof were specifically detected by anti-HA in Western blot analysis. Following treatment with PIs, both Ub^G76V^MelanA-SL and Ub^G76V(K0)^MelanA-SL displayed a ladder of bands with reduced mobility, showing that HA-Ub molecules were covalently attached to those variants. Additionally a high-molecular weight smear could be detected, which most probably represents polyubiquitin-chains which consist of several ubiquitin molecules that are linked with each other via K48 and are covalently attached to one of the remaining lysine residues within the MelanA part of the fusion protein (Fig. 3B). In the absence of PIs neither Ub^G76V^MelanA-SL nor Ub^G76V(K0)^MelanA-SL could be detected in the Western blot. In contrast, MelanA-SL shows ubiquitinated species in the absence and presence of PIs, most probably representing polyubiquitin-chains, which consist of several ubiquitin molecules that are linked with each other via K63 and are also covalently attached to a lysine residue within MelanA-SL. This modification is crucial for the transport of the protein throughout the trans-Golgi network, as shown previously by others [33], and does not represent a signal for proteasomal degradation.

Flow cytometry revealed that cells expressing Ub^G76V(K0)^MelanA-SL or Ub^G76V^MelanA-SL displayed a two-fold increase in the amount of H2-K^b^-SL complexes at the cell surface when compared to cells expressing the original MelanA-SL (Fig. 3 C+D). These results demonstrate that the reduced stability as well as the increased MHC-I antigen presentation of Ub^G76V^MelanA-SL are independent of the Lys residues within the fused Ub moiety.

### Only one lysine residue, independent of its position, can target Ub^G76V(K0)^MelanA-SL into the UPS

As the Lys residues within the fused Ub are dispensable for an efficient proteasomal degradation of Ub^G76V^MelanA-SL, we wanted to know if a specific Lys residue within the MelanA-SL fusion part is polyubiquitinated instead. The luminal N-terminal part of MelanA is followed by a transmembrane domain and the cytosolic C-terminal region [27]. *In silico* analysis using the SOSUI algorithm [34] revealed that fusion of Ub^G76V^ to the N-terminus of MelanA-SL does not affect its topology (Fig. 4A). The Lys residues at positions 19 (introduced by the SL-motif), 24 and 25 are predicted to be located in the lumen, whereas those on positions 70, 95, 101 and 116 are cytosolic (Fig. 4A). Individual mutation of each of the seven Lys residues in the context of Ub^G76V(K0)^MelanA-SL (K24, K25, K70, K95, K101, K116) to Arg had no influence on the stability or MHC-I antigen presentation (data not shown). This indicates that there is no unique, specific ubiquitination site within MelanA-SL.

**Figure 4:** Only one lysine residue, independently of its position, can target Ub^G76V(K0)^MelanA-SL into the UPS. (**A**) Schematic depiction of Ub^G76V(K0)^MelanA-SL in the ER membrane. The Lys residues within MelanA-SL are marked in red. (**B+C**) HeLa cells were transiently transfected with expression plasmids coding for MelanA-SL, Ub^G76V^MelanA-SL, Ub^G76V(K0)^MelanA-SL or variants thereof harboring cumulative Lys to Arg mutations (**B**) from the C- to the N-terminus or (**C**) from the N- to the C-terminus. Cells were treated with PIs or DMSO for 4 h. Whole cell lysates were analyzed by Western blot. As a loading control, the Western blot was reprobed using an anti-β-actin Ab. (**D**) Depiction of the mean fluorescence intensity (MFI) of the 25D1.16 staining of six independent experiments using MelanA-SL and Ub^G76V(K0)^MelanA-SL^K19only^. The statistical analysis was performed using the paired two-tailed student's t-test (_***_p<0.0001). (**E**) Following transient transfection, HeLa cells expressing MelanA-SL, Ub^G76V^MelanA-SL, Ub^G76V(K0)^MelanA-SL or Ub^G76V(K0)^MelanA-SL variants harbouring only one of the lysine residues within MelanA were treated with PIs or DMSO for 4 h prior to lysis. Whole cell lysates were analyzed by Western blot. As a loading control, the Western blot was reprobed using an anti-β-actin Ab.

The ER-resident E3 Ub ligases identified so far have their catalytic RING domain at cytosolic face of the ER membrane [18]. We therefore hypothesized that one of the cytosolic Lys residues of Ub^G76V(K0)^MelanA-SL should be polyubiquitinated. To test this assumption, all Lys residues within Ub^G76V(K0)^MelanA-SL were successively mutated to Arg from the C- to the N-terminus. The Lys residue at position 19 was not exchanged, as it is essential for the recognition of H2-K^b^-SL complexes by the mAb 25D1.16. Mutation of Lys residues 116-70 had no effect on the stability of Ub^G76V(K0)^MelanA-SL (Fig. 4B). Additional mutations of the Lys residues 24/25 mildly reduced the enhanced degradation, though not to wt levels (Fig. 4B). This indicates that cytosolic Lys residues are dispensable for the augmented proteasomal degradation and antigen presentation of Ub^G76V(K0)^MelanA-SL.

Successive mutation of the Lys residues within Ub^G76V(K0)^MelanA-SL from the N- to the C-terminus had very similar effects on protein levels as shown by Western blot analysis (Fig. 4C). The exchange of Lys residues for Arg, starting at position 24 up to 101 had no, or only marginal effects on protein stability. Additional mutation of the Lys residue at position 116 attenuated the rapid degradation, but again not to wt levels. Moreover the MHC-I antigen presentation of Ub^G76V(K0)^MelanA-SL with only one lysine residue (K19) is still highly significantly enhanced when compared to the wt (Fig. 4D).

These results indicate that there is no specific ubiquitination site within Ub^G76V^MelanA-SL, neither in the C-terminal nor in the N-terminal region, that can drive Ub^G76V^MelanA-SL into the UFD-pathway.

We have shown above that the Lys residue at position 19 of MelanA is sufficient to induce its proteasomal degradation (Fig. 4 B+C). We now want to analyze if this is also valid for the other lysine residues along MelanA. Therefore we created mutants where all lysine residues of MelanA within the Ub^G76V(K0)^MelanA-SL fusion protein were exchanged to alanine, except one. The mutants were called Ub^G76V(K0)^MelanA-SL^K24/25only^, Ub^G76V(K0)^MelanA-SL^K70only^, Ub^G76V(K0)^MelanA-SL^K95only^, Ub^G76V(K0)^MelanA-SL^K101only^ and Ub^G76V(K0)^MelanA-SL^K116only^.

Western blot analysis of the whole cell lysates show that the stability of these mutants is only slightly increased. Nevertheless, after treatment with PIs, all mutants are obviously stabilized, indicating that they are still rapidly degraded by the 26S proteasome (Fig. 4E).

Taken together, this cumulative data clearly illustrate that one position independent lysine residue is sufficient to target Ub^G76V(K0)^MelanA-SL into the UPS.

### Mutation of all Lys residues within Ub^G76V^MelanA-SL abrogates its entry into the UFD-pathway

It has been shown previously that also Ser, Thr or Cys residues can be ubiquitinated [1]. To exclude that Ub^G76V(K0)^MelanA-SL is targeted for proteasomal degradation by such atypical polyubiquitination or independently of polyubiquitinylation [35], we mutated all Lys residues within Ub^G76V(K0)^MelanA-SL to Arg (Ub^G76V(K0)^MelanA^(K0)^-SL). Western blot analysis of whole cell lysates demonstrates that the steady-state protein levels of Ub^G76V(K0)^MelanA^(K0)^-SL and MelanA-SL are similar, revealing that the enhanced proteasomal degradation is completely abolished when all Lys residues are mutated. In addition, no ubiquitinated adducts were detectable and the mutant did not further respond to the treatment with PIs (Fig. 5).

**Figure 5:** Mutation of all Lys residues within Ub^G76V^MelanA-SL abrogates its entry into the UFD-pathway. Following transient transfection, HeLa cells expressing MelanA-SL, Ub^G76V^MelanA-SL, Ub^G76V(K0)^MelanA-SL or Ub^G76V(K0)^MelanA^(K0)^-SL were treated with PIs or DMSO for 4 h prior to lysis. Whole cell lysates were analyzed by Western blot. As a loading control, the Western blot was reprobed using an anti-β-actin Ab.

This result clearly shows that the presence of at least one Lys residue is required to target Ub^G76V(K0)^MelanA-SL for degradation by the 26S proteasome.

### Ub^G76V^MelanA-SL and Ub^G76V(K0)^MelanA-SL are degraded via the ERAD pathway

We have shown above that upon proteasome shut-down, the transmembrane protein Ub^G76V^MelanA-SL accumulates in cytosol (Fig. 2). This suggests that the degradation of the Ub^G76V^MelanA-SL fusion protein follows the ERAD pathway, which includes the retranslocation of ER-resident proteins into the cytosol for destruction by the 26S proteasome. To test this hypothesis, we used the potent and specific inhibitor of the ERAD pathway, Eeyarestatin 1 (Eey1; [36]), which inhibits protein retranslocation by targeting both the ER membrane and the AAA-ATPase VCP/p97 [37], [38].

Western blot analysis of whole cell lysates revealed that in the absence of PIs and Eey1, Ub^G76V^MelanA-SL and Ub^G76V(K0)^MelanA-SL are efficiently degraded (Fig. 6 A, lanes 1–3). Treatment with 40 µM Eey1 for 4 h (Fig. 6 A, lanes 4–6) caused the accumulation to protein levels comparable to those obtained after addition of PIs alone (Fig. 6 A, lanes 7–9) or in combination with Eey1 (Fig. 6 A, lanes 10–12).

**Figure 6:** Ub^G76V^MelanA-SL and Ub^G76V(K0)^MelanA-SL are degraded via the ERAD-pathway. After transient transfection, HeLa cells expressing MelanA-SL, Ub^G76V^MelanA-SL or Ub^G76V(K0)^MelanA-SL (**A**) or GFP, Ub^G76V^GFP or UbMGFP (**B**) were treated with PIs or DMSO in the presence or absence of the ERAD-inhibitor Eey1 for 4 h. Whole cell lysates were analyzed by Western blot. As a loading control, the Western blot was reprobed using an anti-β-actin Ab. (**C**) HeLa cells were transiently transfected with MelanA-SL or Ub^G76V^MelanA-SL and treated with PIs or DMSO for 4 h or ExoA for 18 h. Whole cell lysates were analyzed by Western blot. As a loading control, the Western blot was reprobed using an anti-β-actin Ab. To document the uptake of ExoA the Western blot was stained with an anti-ExoA Ab. (**D**) 24 h after transient transfection of MelanA-SL or Ub^G76V^MelanA-SL in HeLa-K^b^ cells, ExoA was added for 18 h. After acid wash a fraction of the cells was harvested (0 h). The other part was further incubated for 4 h in complete RPMI 1640 medium with or without ExoA. H2-K^b^-SL complexes presented on the surface of MelanA-positive cells were quantified by flow cytometry using 25D1.16-APC. The mean fluorescence intensity (MFI) of the 25D1.16 staining of four independent experiments is depicted. Bars represent mean ± SD.

Besides the ERAD pathway, VCP/p97 is also an important component of the UFD pathway [21]. To exclude unspecific inhibitory effects of Eey1 on VCP/p97 or the proteasome, we analyzed the influence of the ERAD inhibitor on the already characterized cytosolic substrate of the UFD pathway, Ub^G76V^GFP [4], [12]. HeLa cells were transfected with expression constructs coding for GFP, Ub^G76V^GFP or the cleavable Ub fusion UbMGFP. Following cleavage of Ub, the latter corresponds to wt GFP. Ub^G76V^GFP can be efficiently rescued from proteasomal degradation by the addition of PIs (Fig. 6 B, lanes 2 and 8), while treatment with Eey1 had no influence (Fig. 6 B, lane 5). The protein levels of GFP or UbMGFP were neither influenced by PIs, Eey1 nor the combination of both. Based on this observation, we conclude that it is unlikely that the stabilizing effects of Eey1 on Ub^G76V(K0)^MelanA-SL are due to unspecific inhibitory effects on the UFD pathway or the UPS.

To confirm the results obtained for Eey1 we also used another specific inhibitor of the ERAD pathway, Exotoxin A (ExoA), as described previously [39], [40]. Western blot analysis of whole cell lysates revealed that in the absence of PIs and ExoA, Ub^G76V^MelanA-SL is degraded by the 26S proteasome. Treatment with ExoA blocked the degradation of Ub^G76V^MelanA-SL and caused an accumulation of the protein similar to the phenomenon obtained after addition of PIs (Fig. 6 C). To verify that the exogenously added ExoA is indeed incorporated into the cell, the Western blot was reprobed and ExoA was detected after staining with an anti-ExoA antibody.

It was shown previously that epitopes generated for MHC-I presentation from an ER-targeted protein are presented by MHC-I molecules without being processed by the ERAD pathway [40]. To analyse if this is also the case for Ub^G76V^MelanA-SL, we measured the H2-K^b^-SL presentation following treatment with ExoA. To remove the H2-K^b^-SL complexes from the cell surface, which had already been loaded before treatment with ExoA, an acid wash of cells was performed and 4 hours later the H2-K^b^-SL presentation was measured. While the acid wash removed most of the H2-K^b^-SL-complexes from the cell surface (Fig. 6D; time point 0), four hours later the MHC-I antigen presentation of Ub^G76V^MelanA-SL treated with ExoA was clearly reduced almost to wt levels (Fig. 6D). The total amount of H2-K^b^-molecules at the cell surface was not influenced by the treatment with ExoA (data not shown).

These results show that Ub^G76V^MelanA-SL is degraded via the ERAD pathway which is crucial for an efficient MHC-I antigen presentation of SL epitopes derived from this ER resident protein.

## Discussion

We show here that a stable fusion of Ub^G76V^ to its luminal N-terminus converts the transmembrane model protein MelanA-SL into a substrate for both the UFD and the ERAD pathway. In contrast to the current working model of the UFD pathway, the degradation and MHC-I antigen presentation of Ub^G76V^MelanA-SL were independent of Lys residues within the fused Ub moiety, but dependent on the presence of the primary sequence of Ub and at least one position independent Lys residue within the entire fusion protein.

Our finding that N-terminal in frame fusion of Ub^G76V^ to MelanA has enhancing effects on its proteasomal degradation and MHC-I antigen presentation further underlines results obtained for a number of cytosolic [4], [5], [6], [7], [8], but only few membrane proteins [9], [10] characterized in previous studies. In addition to that, we observed that neither the integrity of Lys-29 and Lys-48, nor any other Lys residue within the Ub fusion part of Ub^G76V^MelanA-SL were essential to induce rapid proteasomal degradation of the fusion protein. Although, to our knowledge, this requirement for Lys residues has not been studied for transmembrane substrates of the UFD pathway so far, this result is in contrast to findings reported for cytosolic UFD substrates [6], [22], [41].

Alterations in subcellular localization have been shown to enhance the proteasomal degradation and thus the MHC-I antigen presentation of certain proteins [30], [31]. Therefore, we confirmed by immunocytochemistry and cellular fractioning (Fig. 2) that the introduction of SL, as well as the Ub^G76V^ fusion, did not interfere with the insertion of MelanA into the ER membrane, as suggested by *in silico* prediction. Following inhibition of proteasomal activity, Ub^G76V^MelanA-SL accumulated in the ER, but also in the cytoplasm. This indicates that at least a fraction of the protein is degraded via the ERAD pathway. Indeed, degradation of the transmembrane UFD model substrate Ub^G76V^MelanA-SL, but not the soluble UFD substrate Ub^G76V^GFP [4], [12], was inhibited by the VCP/p97-specific inhibitor Eey1 which has no influence on the catalytic activity of the 26S proteasome [36]. Addition of PIs alone or in combination with Eey1, however, stabilized Ub^G76V^MelanA-SL more effectively than treatment with Eey1 alone. Though, alternative p97/VCP- and ubiquitination-independent routes to exit the ER have been reported [17], this effect might rather be explained by proteasomal degradation of a fraction of Ub^G76V^MelanA-SL that has not been inserted into the ER membrane yet, or has already been extracted from the ER membrane prior to addition of Eey1. In addition, it cannot be completely ruled out that the concentration of Eey1 used in our experiments might be insufficient for complete inhibition of the retranslocation from the ER to the cytosol. To further substantiate the results obtained with Eey1 we used as another inhibitor of the ERAD pathway ExoA as described before [39], [40]. ExoA stabilizes Ub^G76V^MelanA-SL in the same way as Eey1 providing another proof that Ub^G76V^MelanA-SL is indeed degraded by the ERAD pathway (Fig. 6C). It was shown recently by Schlosser *et al.* that the generation of epitopes of the prostate carcinoma antigen (PSCA) presented by MHC-I molecules completely occurs in the cytoplasm before the protein is inserted into the ER and thus without any involvement of the ERAD pathway [40]. In contrast, for the generation of epitopes derived from Ub^G76V^MelanA-SL the ERAD pathway is crucial, as the blockade of this pathway by the addition of ExoA clearly reduces its MHC-I antigen presentation almost to wt levels (Fig. 6D).

It is also legitimate to speculate from our results that there might be a different mechanism in targeting cytosolic and transmembrane UFD substrates for proteasomal degradation. According to the UFD model for cytosolic substrates, the N-terminal Ub fusion part serves as attachment side for polyubiquitin chains [5], [6], [42]. For transmembrane substrates, the fused Ub moiety seems to be a signal for VCP-mediated retranslocation of the fusion protein back to the cytosol. One possible scenario is that after retranslocation cellular factors are recruited, which then scan the whole fusion protein for at least one remaining lysine residue and thus mediate the polyubiquitination signal. Currently it is not clear, if at that point the Ub moiety is still necessary for triggering position independent polyubiquitination, as the folding of the protein might be different after retranslocation. For cytosolic UFD substrates it has been shown previously that the E3-ligase TRIP12 plays an important role in the attachment of polyubiquitin chains [14]. It remains to be investigated if TRIP12 also plays a role in polyubiquitination of transmembrane UFD substrates. Another scenario could be that ubiquitination starts at the cytosolic face of the fusion protein, even prior to retranslocation. This possibility would correspond to the observation that polyubiquitination is required for the retranslocation of some ER resident proteins back to the cytosol [43].

It has been shown that polyubiquitination on Ser or Thr residues can signal for degradation via the ERAD pathway [1]. Moreover, some proteins can even be degraded by the proteasome in absence of polyubiquitination [35]. The proteasomal degradation of Ub^G76V^MelanA-SL, however, was dependent on the presence of at least one Lys residue within the fusion protein. When all lysine residues were removed, the degradation of MelanA was completely abolished and the mutant did not further respond to the treatment with PIs (Fig. 5).

In comparison with the Ub^G76V^MelanA-SL where all lysine residues were conserved, in the presence of only one lysine residue, the degradation as well as the MHC-I presentation of Ub^G76V^MelanA-SL were only mildly reduced (Fig. 4). These findings strongly suggest that canonical Lys-linked polyubiquitination is the major, if not the only way to target Ub^G76V^MelanA-SL for proteolysis by the 26S proteasome.

Interestingly, the enhanced degradation and MHC-I antigen presentation of Ub^G76V^MelanA-SL was independent of the Lys residue's location within the protein (Fig. 4). This indicates that polyubiquitination might not only occur at Lys residues located at the cytoplasmic face of the ER, as observed before for MelanA wt [44], but also at a Lys residue within the luminal N-terminus of Ub^G76V^MelanA-SL. To date, however, all Ub E3 ligase activity has been mapped to the cytoplasmic face of the ER [18].

There are mainly two different explanations for this paradigm: First, there might be a so far unpresented ER-resident E3 ligase that has at least its catalytic domain orientated towards the lumen. Second, Ub^G76V^MelanA-SL might be partially extracted from the ER prior to polyubiquitination. The second hypothesis is strengthened by the observation that Ub^G76V^MelanA-SL does exist in the membrane fraction in an ubiquitinated manner, indicating that the polyubiquitination of this protein occurs prior to the retranslocation into the cytosol (Fig. 2C). A fraction of Ub^G76V^MelanA-SL, however, accumulated in the cytoplasm after the inhibition of the proteasome (Fig. 2), underlining that the protein is, at some point, extracted from the ER membrane. This is consistent with the notion that polyubiquitination is a prerequisite for the segregation of most ERAD substrates [43].

VCP/p97 has been implicated in the UFD pathway in yeast [21], [23]. In addition, three components of the UFD pathway, namely Ufd1, Ufd2 and Ufd3 have been shown to act in the ERAD pathway by interacting with VCP/p97 (reviewed in [45]). However, the detailed entwinement of the UFD and ERAD pathways and the role of their components for the degradation are still awaiting investigation.

Another open question remaining is how the N-terminal Ub moiety is recognized in the ER lumen and targeted to the ERAD machinery. VCP/p97 is known to interact with a variety of cofactors [45], many of which have Ub binding domains (UBDs; [46], [47]). Therefore, one possibility might be that a cellular protein with an UBD binds to VCP and is thereby recruited to the ER membrane following recognition of the fused Ub moiety. UBDs most commonly recognize a hydrophobic patch composed of residues Leu-8, Ile-44 and Val-70 of Ub [46], [47]. Alternatively, the regions around Ile-36 or Asp-58 of Ub have been described as interaction sites [46], [47]. Nevertheless, the proteins involved in the ERAD and UFD pathways that recognize such Ub fusion proteins, their UBD and the residues within Ub critical for that recognition remain to be identified.

The activation of naive cytotoxic CD8^+^ T-cells is mainly based on two pathways, the direct-presentation and the cross-presentation pathway [48]. Both include the presentation of antigenic peptides on the cell surface loaded onto MHC-I molecules but the source of these peptides is quite different. Cross presentation on the one hand requires stable antigens to induce an efficient T-cell response [48], [49], [50]. It was shown recently that after DNA vaccination with a recombinant vaccinia virus the CD8^+^ T-cell response is strongly induced in the presence of stable antigens [51]. On the contrary, DNA vaccination studies also showed that especially instable antigens can cause a better T-cell response [7], [31], [52], [53]. This is in concert with the observation that the main source of antigens for direct MHC-I presentation are rapidly degraded proteins, the so called defective ribosomal products (DRiPs) [54]. As both presentation pathways can efficiently elevate the T-cell response against specific antigens, even though by different modes of action, they can equally be applied in the development of vaccination strategies.

Taken together, we get here two important findings: First, we could clearly enhance the immunogenicity of the important tumor antigen MelanA. As this antigen is used in DC vaccination, our findings could be helpful to improve the vaccination against malignant skin cancer. Second, we have demonstrated that fusion of an N-terminal mono-Ub to a transmembrane protein results in targeting of the protein to the UPS independently of Lys residues within the Ub fusion part and in the presence of at least only one position independent Lys residue. This illustrates a new concept for the UFD as such a mechanism has never been shown before.

## Materials and Methods

### Plasmid constructs

The sequence coding for the SL epitope, corresponding to amino acids 257–264 of ovalbumin, was introduced into the MelanA-coding sequence using a unique Bst EII site and oligonucleotides BstEII-SL-fw (5′-GTT ACT CGA TCA TCA ACT TCG AAA AGC TAG-3′) and BstEII-SL-rw (5′- GTA ACC TAG CTT TTC GAA GTT GAT GAT CGA-3′). For the construct pUb^G76V^MelanA-SL, overlapping DNA fragments were fused by PCR using the oligonucleotides EcoRI-UbV fw (5′-TGC TGG AAT TCG CCG CCA CCA TGC AGA TCT TCG-3′), UbV rev (5′-GCA TCT TCT CTT GGC ATC ACC CCC CTC AAG CG-3′), MelanA-UbV fw (5′-TTG AGG GGG GTG ATG CCA AGA GAA GAT GCT CAC-3′), MelanA-XbaI rev (5′-GAT GCA TGC TCG AGG TAA TTA AGA ATG TGC AGC-3′) and cloned into pcDNA3.1 using EcoRI and XbaI. Point mutations were introduced by site directed mutagenesis using the Quikchange kit (Stragene) and following oligonucleotides: UbV K6R fw (5′-GAT CTT CGT GAG GAC CCT GAC CGG C-3′), UbV K6R rev (5-′GCC GGT CAG GGT CCT CAC GAA GAT C-3′), UbV K11R fw (5-′CCC TGA CCG GCA GGA CCA TCA CCC TGG-3′), UbV K11R rev (5-′CCA GGG TGA TGG TCC TGC CGG TCA GGG-3′), UbV K27R fw (5-′CCA TCG AAA ATG TGA GGG CCA AGA TCC AGG-3′), UbV K27R rev (5-′CGA AAA TGT GAA GGC CAG GAT CCA GGA TAA AGA AGG-3′), UbV K29R rev (5-′CCT TCT TTA TCC TGG ATC CTG GCC TTC ACA TTT TCG-3′), UbV K33R fw (5-′GCC AAG ATC CAG GAT AGA GAA GGC ATC CCC CC-3′), UbV K33R rev (5-′GGG GGG ATG CCT TCT CTA TCC TGG ATC TTG GC-3′), UbV K48R fw (5-′GCT CAT CTT TGC AGG CAG ACA GTT GGA AGA TGG C-3′), UbV K48R rev (5-′GCC ATC TTC CAA CTG TCT GCC TGC AAA GAT GAG C-3′), UbV K63R fw (5-′CAA CAT CCA GAG AGA GTC GAC CCT GCA TCT GG-3′), UbV K63R rev (5-′CCA GAT GCA GGG TCG ACT CTC TCT GGA TGT TG-3′), MelanA K19R fw (5-′CGA TCA TCA ACT TCG AAA GAC TAG GTT ACC CC-3′), MelanA K19R rev (5-′GGG GTA ACC TAG TCT TTC GAA GTT GAT GAT CG-3′), MelanA K24/25R fw (5-′GGT TAC CCC AGA AGA GGG CAC GGC C-3′), MelanA K24/25R rev (5-′GGC CGT GCC CTC TTC TGG GGT AAC C-3′), MelanA K70R fw (5-′CCT TGA TGG ATA GAA GTC TTC ATG TTG GC-3′), MelanA K70R rev (5-′GCC AAC ATG AAG ACT TCT ATC CAT CAA GG-3′), MelanA K95R fw (5-′CGG GAC AGC AGA GTG TCT CTT CAA G-3′), MelanA K95R rev (5-′CTT GAA GAG ACA CTC TGC TGT CCC G-3′), MelanA K101R fw (5-′CTC TTC AAG AGA GAA ACT GTG AAC CTG TGG-3′), MelanA K101R rev (5-′CCA CAG GTT CAC AGT TTC TCT CTT GAA GAG-3′), MelanA K116R fw (5-′CCT GCT TAT GAG AGA CTC TCT GCA GAA CAG TCA CC-3′), MelanA K116R rev (5-′GGT GAC TGT TCT GCA GAG AGT CTC TCA TAA GCA GG-3′).

### Cell culture

HeLaSS6 cells were cultured in DMEM supplemented with 10% (v/v) inactivated FCS, 2 mM L-glutamine, 100 U/ml penicillin and 100 µg/ml streptomycin. For HeLa-K^b^ cells, 1 mg/ml G418 was added. Inhibitors LC (5 µM; Boston Biochem), MG-132 (20 µM, Sigma) or Eey1 (40 µM; Tocris) were added for 4 h. ExoA (10 µg/ml; Calbiochem) was added for 18 h.

### Western blot

Cells were lysed in RIPA (50 mM Tris-HCl [pH 7.4], 150 mM NaCl, 1% [v/v] Nonidet P-40, 0.5% [w/v] sodium deoxycholate, 0.1% [w/v] SDS, supplemented with 1 mM PMSF, 5 mM N-ethylmaleimide, 20 µM MG-132 and complete protease inhibitor mixture (Roche)). Proteins were separated by SDS-PAGE, blotted onto PVDF membranes (GE Healthcare) and probed with following Abs prior to ECL detection: monoclonal anti-MelanA (Novocastra), monoclonal anti-GFP (Roche), monoclonal anti-ß-actin (Sigma), polyclonal anti-ExoA (Sigma) and monoclonal anti-Hsp90 (Santa Cruz).

### Quantitative RT-PCR analysis

HeLa cells were transiently transfected with expression plasmids that code for MelanA-SL or Ub^G76V^MelanA-SL respectively. 24 h post transfection the total RNA was extracted using the RNeasy Mini Kit (Quiagen) and its quality and quantity was assessed using the BioPhotometer plus (Eppendorf). The qRT-PCR analysis was conducted using the SuperScript®III Platinum® SYBR® Green One-Step qRT-PCR Kit (Invitrogen) according to the manufacturer's instruction. The primer sequences for MelanA-SL were as follows: forward 5′- GGA TCG GCA TCC TGA CAG TGA TC -3′ and reverse 5′- GCA TTG GGA ACC ACA GGT TCA CAG -3′. Each sample was amplified in duplicate and normalized for the housekeeping gene GAPDH. The quantitative RT-PCR was conducted using the Abi 7500 PCR machine (Applied Biosystems).

### Immunoprecipitation

Following coexpression of MelanA-SL and variants thereof with HA- tagged Ub, MelanA-SL contained in ∼800 µg whole cellular proteins was precipitated from the whole cell lysates using anti-MelanA Ab prebound to protein G-Sepharose. Cells were lysed in RIPA (50 mM Tris-HCl [pH 7.4], 150 mM NaCl, 1% [v/v] Nonidet P-40, 0.5% [w/v] sodium deoxycholate, 0.1% [w/v] SDS, supplemented with 1 mM PMSF, 5 mM N-ethylmaleimide, 20 µM MG-132 and complete protease inhibitor mixture (Roche). The Western blot analyses were conducted as described before.

### Flow cytometry

For detection of H2-K^b^-bound SL-epitope, cells were stained with the allophycocyanin (APC)-conjugated 25D1.16 mAb (eBioscience) diluted 1∶100 in FACS buffer (5% [v/v] FCS, 0.02% [v/v] NaN_3_ in PBS). For detection of total H2-K^b^ molecules, cells were incubated with hybridoma cell culture supernatant containing the mAb B8-24-3 [55], followed by staining with secondary Alexa 647-conjugated anti-mouse Ab (Invitrogen). For intracellular MelanA staining, cells were permeabilized using Cytofix/Cytoperm (BD Bioscience). MelanA was detected by staining with an anti-MelanA mAb (Novocastra; 1∶25), followed by staining with Alexa 647-conjugated anti-mouse Ab (1∶100), both diluted in Perm/Wash buffer (BD Bioscience). Flow cytometry was performed on a FACSCalibur using CellQuest software (BD Bioscience). Data were analyzed by using the FACS Express V3 software (De Novo Software).

### Acid Wash

HeLa-K^b^ cells were transiently transfected with expression plasmids that code for MelanA-SL or Ub^G76V^MelanA-SL respectively. 24 h later ExoA was added for 18 h. Subsequently newly H2-K^b^-SL-complex formation at the cell surface was followed by flow cytometry after an acid wash procedure as described previously [56]. Cells were harvested right after the acid wash (time point 0) and after 4 hours of incubation in complete RPMI 1640 with and without ExoA and stained for FACS analysis as described above.

### Immunofluorescence microscopy

Cells were fixed in 3% (w/v) paraformaldehyde and permeabilized using 0.1% (v/v) TritonX-100 in PBS. MelanA and the TGN were detected using a mouse anti-MelanA Ab (Novocastra) and a rabbit anti-TGN46 Ab (Abcam), respectively, followed by staining with secondary Alexa488-conjugated anti-mouse and Alexa647-conjugated anti-rabbit Abs (Invitrogen), respectively. The nucleus was visualized by staining with DAPI. Images were obtained using a Leica TCS SP5 confocal microscope with the 63× objective and analyzed by Adobe Photoshop software.

### Cell fractioning

The plasma membrane was permeabilized using 20 µM digitonin as described previously [32]. After centrifugation, the supernatant, containing cytosolic proteins and the pellet, including proteins associated with intracellular membranes, were analyzed by Western blot as indicated.

For the isolation of ER resident proteins an ER isolation kit (Sigma) was used according to the manufacturer's instruction. The ER fraction was analyzed by Western blot as indicated.

### Statistical analysis

Statistical analysis was performed using the Graph Pad Prism software. P-values were calculated by a paired two-tailed student's t-test after confirming that the measured values followed the Gaussian distribution (Kolmogorov-Smirnov)
